# Investigating Subtypes of Motor Skills and Activities of Daily Living among Young Children with Motor Delay

**DOI:** 10.1155/2023/4031372

**Published:** 2023-06-15

**Authors:** Keisuke Irie, Kohei Mukaiyama, Reika Yamashita, Hala Zeidan, Anuradhi Bandara, Momoko Nagai-Tanima, Tomoki Aoyama

**Affiliations:** ^1^Department of Occupational Therapy, Human Health Sciences, Graduate School of Medicine, Kyoto University, Kyoto, Japan; ^2^Department of Physical Therapy, Human Health Sciences, Graduate School of Medicine, Kyoto University, Kyoto, Japan; ^3^Ecold Inc., Osaka, Japan

## Abstract

The purpose of this study was to classify preschool children into subtypes based on motor skills and to characterize the activities of daily living for each subtype. The subjects were 45 preschool children whose scores on the Movement Assessment Battery for Children-Second Edition (MABC-2) and the Functional Independence Measure for Children (WeeFIM) were measured. The fine score and gross score were calculated from the MABC-2, and a cluster analysis was performed. The difference between the fine score and the gross score was evaluated for each subtype, and multiple comparisons among subtypes were performed for the fine, gross, and WeeFIM scores. Subtype analysis showed that the fine score was significantly lower than the gross score for subtype I (*p* < 0.001), and the gross score was significantly lower than the fine score for subtype III (*p* = 0.018). Subtype II had a significantly lower score than subtype I and subtype III (*p* < 0.001). Children with subtype II had more difficulty dressing movements and less communication skills than subtype III (*p* < 0.05). Classification into three subtypes according to motor ability and some of the characteristics of ADLs were identified.

## 1. Background

Developmental coordination disorder (DCD) is a common neurodevelopmental disorder that affecting approximately 5%–6% of school-aged children [1]. The American Psychiatric Association defines DCD as a significant difficulty in learning motor skills without sensory, intellectual, or neurological impairment. Children with DCD may be described as “clumsy” because their motor coordination is below the level expected for their age [2]. Movement disorders are prominent from early childhood and often continue into adolescence and adulthood [3]. Children with DCD may have difficulty with either gross or fine motor coordination or both, which may affect their academic performance and activities of daily living (ADLs) such as eating, dressing, and grooming [2, 4]. It is well known that DCD is associated with reduced physical activity [5, 6]. In addition to that, difficulties with peer relations [7], low self-esteem [8], anxiety [9], and depression [10] are frequently reported psychosocial problems in the DCD population.

Clumsiness in children with DCD has been attributed to differences in brain activity compared to typically developing (TD) children. Neural activity in multiple brain regions, including the frontal lobe, parietal lobe, basal ganglia, and cerebellum, has been found to be reduced [11, 12]. However, the symptoms of DCD children may vary widely because the areas of reduced brain function vary from one child to another. In order to effectively address the impaired motor skills exhibited by children with DCD, it is important to divide them into distinct subtypes based on similar characteristics. Previous research studies used the various psychomotor and clinical characteristics to identify subtypes of DCD [13–25]. For example, Dewey and Kaplan [15] used balance, bilateral coordination, upper limb coordination, gestures, and motor sequencing as measurements and identified four subtypes. Previous studies focused on subtypes of DCD differed in many points, including sample size, assessment procedures, instrumentation, statistical methods, and the number of identified subtypes. However, previous research supports the concept that subtypes and heterogeneous clinical presentations exist among children with DCD. Furthermore, many studies agree on the existence of subtypes with generalized gross and fine motor movements [15, 18, 20, 21, 24, 25]. In general, a technique called cluster analysis has been used for subtype classification [20, 22]. Previously, DCD subtype studies reported three to six clusters of DCD emerging from different combinations of variables [14, 15, 18, 20–22].

The Movement Assessment Battery for Children-Second Edition (MABC-2) is used worldwide [1, 26], especially to test for one of the diagnostic criteria of DCD according to the Diagnostic and Statistical Manual of Mental Disorders-V (DSM-V) [2]. A Japanese version of the MABC-2 exists and is of comparable utility [27, 28]. Most studies of DCD have been conducted on children aged 6 years and older, and few have been conducted on preschoolers [16, 29]. This is due to the potential for variability in MABC-2 test results in preschool children, which makes diagnosis difficult. However, it is worthwhile to conduct further research on children younger than 6 years of age, as early support has recently been reported to be necessary [30]. Furthermore, with the lowering of the age range for the MABC-2 from 4 to 3 years in 2007 [31, 32], this test battery may be increasingly useful in the motor assessment of children in the early stages. Gross motor skills are those that coordinate the upper and lower limbs and trunk to produce large movements. In contrast, fine motor skills are those that produce small, precise movements centered on the fingers [33]. Children with DCD may have difficulties in a broad range of motor-based ADL, including mobility, personal hygiene, eating, dressing (managing buttons and zippers and tying shoelaces), and toileting [34–36]. Delays in ADL learning, poor ADL performance, and less frequent participation in ADL are frequently reported problems in children with DCD compared to their typically developing peers [34–37]. Moreover, there is a lack of knowledge about children's specific difficulties in performing and participating in ADL [38]. However, none have simultaneously studied the relationship between different DCD subtypes and ADL. In supporting exercise and daily living, knowing the characteristics of ADL by subtype will help us understand the points we should focus on supporting.

Based on the above, the purpose of this study was to establish a subtype classification of children with motor clumsiness based on fine and gross motor using the MABC-2 and to determine the relationship between these subtypes and ADLs. Four subtypes were assumed: fine motion inferior to coarse motion, coarse motion inferior to fine motion, both fine and coarse motion inferior, and both fine and coarse motion generally good. We hypothesized that the type with poor fine motor skills would be impaired in daily activities requiring coordination of fingers and hands, such as upper body dressing and buttoning and unbuttoning, while the type with poor gross motor skills would be impaired in daily activities requiring mobility and balance skills, such as transferring and moving.

## 2. Methods

### 2.1. Participants

The participants were recruited from developmental support classrooms that provide education and habilitation programs appropriate to the children with a disability booklet. Documents explaining the research plan, the study purpose, and a written consent document were sent to the children and their parents. Those who wished to enrol sent back their written informed consent signed by one of the parents. The recruitment process lasted for approximately two months. Participation criteria were independently mobile preschool children aged 3 to 6 years, and exclusion criteria were those with intellectual disabilities or severe neurological, mental, or physical problems. None of the children with consent for participation had any of these exclusion criteria; thus, 45 participants were included in this study. Measurements were taken in the developmental support classrooms normally used by children. To ensure that the children felt comfortable with the measurements, a familiar teacher was present by their side. This study was approved by the ethical committee of Kyoto University (approval number: R2929).

### 2.2. Procedure

Measurements were taken by one physical therapist who worked in the classroom and knew the children well. First, MABC-2 was first implemented individually. If concentration did not continue or if the child refused, it was administered again at a later date. Thus, all children completed the MABC-2 measurement. Using the raw scores of the subtests included in the MABC-2, we calculated standard scores by expressing the sum of the three MD tests as MD SS, the sum of the two AC tests as AC SS, and the sum of the three BAL tests as BAL SS [32]. The MD test is considered a fine motor task [31] and the AC test [31, 39] and the BAL test as a gross motor task [31]. We distinguished the MD test as children's fine motor skills and the AC and BAL tests as children's gross motor skills. The fine score was set as MD SS, and the gross score was calculated as follows: (AC SS + BAL SS) × 3/5. This is because AC and BAL have 5 tests while MD has only 3 tests. Lower score values indicate lower motor skills. The results of these calculations were used for cluster analysis.

WeeFIM was scored by one occupational therapist who reviewed the children's activities of daily living. All items that could not be verified in the classroom were completed by interviewing the parents.

### 2.3. Measuring Instruments

#### 2.3.1. Movement Assessment Battery for Children-2 (MABC-2)

Motor function was measured using MABC-2 (9780749101732; Pearson Educ. Inc., London, UK), which is targeted at children aged 3–16 years [32]. MABC-2 has different test difficulties for the three age groups, and we used the tests from age band 1, which is for children aged 3 to 6 years. Age band 1 tests consist of three components: manual dexterity (MD), aiming and catching (AC), and balance (BAL). The MD component includes three tasks: a one-hand posting task (posting coins), a timed bimanual assembly task (reading beads), and an untimed drawing task (drawing trail 1). The AC component includes two tasks: throwing an object to a target (throwing a beanbag onto a mat) and catching an object using both hands (catching a beanbag). The BAL component includes three tasks: a static balance task (one-leg balance), two dynamic balance tasks that involve sustained, controlled movements (walking heels raised), and a more explosive action (jumping on a mat). The raw scores of each of these eight tasks were converted to age-adjusted standard scores, and the sum of the latter was considered the MABC-2 total test score. MABC-2 total score was further converted into a percentile rank from 0.1 to 99.9. As shown in Table 1, the percentile rank indicates movement difficulty; the red zone indicates movement difficulty, the amber zone indicates a risk of movement difficulty, and the green zone indicates no movement difficulty. All processes were performed according to the MABC-2 manual [32]. A previous study showed the validity of MABC-2 targeted at Japanese 3–6-year-old children [27].

#### 2.3.2. Functional Independence Measure for Children (WeeFIM)

WeeFIM is an index for evaluating pediatric independence in ADL, which was created based on the Functional Independence Measure (FIM) for adults; it is targeted at nondisabled children aged 6 months to 8 years, children with developmental disabilities aged 6 months to 12 years, and individuals of all ages with developmental disabilities and mental age of less than 7 years [40]. Similar to the FIM, WeeFIM consists of 18 items: 13 exercise items and five cognitive items. All items were rated from 1 to 7 according to their level of independence [40], and the total score of motor items, the total score of cognitive items, and the total score of all items were calculated. The total score ranges between 18 and 126 points, and a high value indicates that the child has a higher degree of independence. The WeeFIM is also a tool that has been tested for reliability and validity for the assessment of ADLs in children [41–43].

### 2.4. Statistical Analyses

The normality of the data was examined using the Shapiro–Wilk test. *K*-means cluster analysis was used in this study to classify children with coordination problems in terms of fine and gross motor skills, using the fine and gross movement scores calculated from MABC-2 component scores. Cluster analysis was employed for subtype classification as in previous studies [15, 18, 20, 21]. In cluster analysis, the cubic clustering criterion (CCC) is calculated, with a higher CCC indicating an optimal number of classifications in the population. The Mann–Whitney *U* test was then performed to examine the differences between the fine and gross scores for each subtype. In addition, differences between subtypes resulting from cluster analysis in age, percentile rank, fine score, and gross score were examined by one-way ANOVA, and the same analysis was performed for WeeFIM scores using the Bonferroni method for post hoc comparisons.

Cluster analysis was performed using JMP Pro 15 (SAS Institute Inc., Cary, North Carolina, USA). Mann–Whitney *U* test and one-way analysis of variance with a Bonferroni correction for post hoc comparison were conducted using IBM SPSS Statistics version 28.0 (IBM Corp., Armonk, NY, USA). Statistical significance was set at *p* < 0.05.

## 3. Results

The CCC is shown in Figure 1, and the optimal number of clusters is three because the highest cluster number is three, excluding the cluster number of one. Cluster analysis based on fine and gross scores classified the children into three subtypes (Figure 2). Tables 2 and 3 show descriptive statistics for each subtype, including total number, percentile rank, and gender. There was no significant difference in age between the subtypes. Subtype analysis showed that the fine score was significantly lower than the gross score for subtype I (*p* < 0.001), and the gross score was significantly lower than the fine score for subtype III (*p* = 0.018). Subtype II had a significantly lower score than subtype I and subtype III (*p* < 0.001), although there was no significant difference between the fine and gross scores (Tables 4 and 5).

The results of the comparison of WeeFIM for each subtype are shown in Table 6. In the exercise domain, subtype II tended to score lower than subtype III in dressing (upper body) (*p* = 0.07), and subtype II scored significantly lower than subtype III in dressing (lower body) (*p* = 0.046). In the cognitive domain, subtype I and subtype II scored significantly lower than subtype III in comprehension and expression (*p* = 0.013 and *p* = 0.026, respectively). Furthermore, in the cognitive subscores, subtype I and subtype II also scored significantly lower than subtype III (*p* = 0.025 and *p* = 0.035, respectively) In the total score, subtype I had a significantly lower total score than subtype III (*p* = 0.033).

## 4. Discussion

In this study, we examined the MABC-2 to subtype children's motor abilities by fine and gross motor and to characterize ADLs for each type. The results of the cluster analysis divided the children into three groups. Furthermore, characteristics of ADLs by type were revealed in the assessment items of dressing movement and cognition.

### 4.1. Subtypes of Fine and Gross Motor Skills

Comparing the difference between the fine and gross scores for each type, the fine score was significantly lower than the gross score for subtype I, and the gross score was significantly lower than the fine score for subtype III. A comparison of percentile ranks showed similar results, with subtype II, subtype I, and subtype III having larger scores in that order. Based on the above, subtype I children are considered to have “significantly worse fine motor activity than coarse motor activity,” subtype children have “both poor fine and coarse motor activity,” and subtype III children have “significantly worse coarse motor activity than fine motor activity.” Furthermore, subtype III children are considered to have good motor function, while subtype I and subtype II children are considered to have possible DCD. Wright and Sugden conducted cluster analysis similar to ours based on the MABC and found that their children could be divided into four groups: children who had difficulty in writing, drawing, and other manual skills; children who had overall impairment; children who needed help in all areas but whose difficulties were not as yet severe; and children who had difficulty in throwing, aiming, and receiving skills [25]. This result is very close to our originally formulated hypothesis. For subtype III in this study, the mean percentile rank is 31.1, and 14 out of 17 children are in the green zone. Although subtype III is significantly poor in coarse motor activity, children with subtype III seem to have relatively good motor function. Therefore, it is likely that the present study included a small number of children with good fine movement skills and much lower levels of gross movement skills. Nakai reported the existence of that group, and another previous study also reported that there were four groups, including a group that was poor in fine movement skills [29]. The difference between the results of the previous studies and our study was the low age range of the participants in our study. As gross movement activities, such as ball-playing, are acquired at an earlier age than fine movement activities, such as buttoning and using scissors [44], children may not have acquired enough fine motor skills at the time of testing. Since the children in this study were as young as 3 to 6 years old, it is likely that fewer children were good at fine motor skills and poor at gross motor skills than in previous studies.

The age difference among the subtypes in the study was not significant. The participants of this study, children aged 3–6 years, are considered a generation whose development is greatly influenced by one year of growth [44]. In addition, boys were more likely than girls to have all types. The sex ratio of children with DCD is 2 : 1 to 7 : 1 [2]. The sex ratio of the participants in this study is consistent with the fact that DCD is more common in boys than girls. These results, taking into account the age and sex ratio, could justify the classification of subtypes in this study.

### 4.2. Performance of ADL According to the Subtype Classification

Comparison of WeeFIM among the types revealed that in the motor items, dressing (upper body) in subtype II tended to be lower than subtype III, and dressing (lower body) in subtype II was significantly lower than subtype III. The average percentile rank in type II was 0.1, the lowest motor function of the three subtypes, while the average percentile rank in subtype III was 31.3, the highest motor function of the three subtypes. Therefore, the comparison of these two subtypes is considered to be close to the comparison of DCD and TD. A previous study reported significant differences in dressing movements between DCD and TD [45], similar to the present results. Furthermore, as subtype III is better at fine movements than at gross movements, good fine motor activity can be considered an additional feature of the difference between subtype II and subtype III. Changing clothes, including the fastening and unfastening of buttons, requires finer motor skills than other tasks, explaining the present results. Contrary to the hypothesis, no differences were found in the subtypes of fine motor activities (eating and toileting activities) and gross motor activities (moving and locomotion). This may be due to the fact that the motor items in the WeeFIM assess their execution regardless of the quality of the activity. Eating and dressing can be performed even if there are spills, etc., if spoons and toothbrushes are provided. In addition, qualitative assessments such as frequency of falls and characteristic gait are not included in the score. For these reasons, differences may not have been recognized. In fact, a previous study similarly reported that there was no significant difference between DCD and TD in items that are part of gross movements, such as transfer and locomotion [46]. Regarding cognitive domains, comprehension, expression, and cognitive subscores in subtypes I and II were significantly lower than those in subtype III. Similarly, a previous study reported lower cognitive scores in DCD than that in TD [46]. Moreover, both fine and gross movement skills help foster language development from infancy to early childhood [47]. Thus, the development of cognitive function, including communication skills, is thought to be related to the development of motor function. Subtypes I and II were found to have lower motor function than subtype III and similarly lower cognitive function. One of the reasons for the small differences in ADL between subtypes was thought to be due to the use of WeeFIM, which has a small change in scores. In the future, utilizing the assessment of motor and process skills [48], which simultaneously assesses the quality and performance of tasks, may help to eliminate the above problem.

Research on subtypes is important for a better understanding of the nature of developmental disabilities. Subtype studies can provide insight into prognosis, specific treatments, and predictions regarding expected health care costs and can be effective in reducing uncertainty about an individual's expected outcome [24, 49, 50]. It is important to identify the specific difficulties that each subtype may face when children are performing and participating in ADL to decide appropriate treatment options. Therefore, this study has a high significance in terms of prioritizing treatment for children who have difficulty in fine and gross motor skills based on the classification results.

This study has several limitations. It is possible that the results of this study were influenced by the size and characteristics of the sample, since the sample size was relatively small (*n* = 45), and the participants were recruited from one school. Additionally, this study targeted children aged 3–6 years. It is not clear if children of other ages would be divided into the same groups. In terms of the analysis, the classification based on the cluster analysis method used here varies among subtypes depending on the participants' performance. Thus, the cut-off values are unknown. Additional studies with bigger sample size and including children above 6 years of age from different schools are needed in the future to decide the correct classification of child subtypes. Besides, since it is necessary to examine the developmental trajectories of children with different subtypes [24], we believe that not only cross-sectional but also longitudinal studies are needed. This study is the first step toward realizing a longitudinal study of subtyping in children.

## 5. Conclusions

This study classified children with motor clumsiness into subtypes based on fine and gross movement skills and investigated the characteristics of ADL in the three subtypes found. Subtype I had “significantly poorer fine movement than gross movement,” subtype II had “both poor fine and gross movements,” and subtype III had “significantly poorer gross movement than fine movement.” Characteristics among the subtypes revealed differences in the performance of ADLs in dressing movements for motor domain and in communication for cognitive domain.

## Figures and Tables

**Figure 1:** Determining the most appropriate number of clusters by the cubic clustering criterion (CCC). CCC is a criterion statistic comparing different models during cluster analysis. The higher the CCC, the better the model will be divided by the cluster.

**Figure 2:** Cluster analysis result based on fine and gross scores. Cluster analysis based on fine and gross scores divided the participants into three groups. Type I had “significantly poorer fine movement than gross movement,” type II had “both poor fine and gross movements,” and type III had “significantly poorer gross movement than fine movement.”

**Table 1:** Children's state and percentile rank with description.

Children's state	Percentile rank	Description
Red zone	At or below the 5th percentile	Denotes a significant movement difficulty
Amber zone	Between the 5th and 15th percentile (inclusive)	Suggests that the child is “at risk” of having a movement difficulty
Green zone	Above the 15th percentile	No movement difficulty noted

**Table 2:** Participant demographics.

Participants	45
Male	35
Female	10
Age (years)	4.7 ± 1.1
Age (months)	62.5 ± 15.1

**Table 3:** Characteristics of each type, total number of children, the number of children per zone, and the number of boys and girls in each subtype.

Subtype	Total number	Percentile rank			Male/female
		Red zone	Amber zone	Green zone	
I	21	21	0	0	15/6
II	7	7	0	0	6/1
III	17	1	2	14	14/3

**Table 4:** Differences between the fine and gross scores among each subtype.

Subtype	Fine	Gross	*p* value
I	13.1.±4.9	19.9 ± 3.6	<0.001^∗^
II	5.9 ± 3.6	7.5 ± 3.7	0.395
III	29.5 ± 6.0	23.9 ± 4.2	0.018^∗^

^∗^ *p* < 0.05.

**Table 5:** Differences among subtypes based on fine score, gross score, age, and percentile rank.

	Subtype			*p* value	*p* value Subtype		
	I	II	III		I-II	I-III	II-III
Fine score	13.1 ± 4.9	5.9 ± 3.6	29.5 ± 6.0	0.000^∗^	0.028^∗^	0.000^∗^	0.007^∗^
Gross score	19.9 ± 3.6	7.5 ± 3.7	23.9 ± 4.2	0.000^∗^	0.001^∗^	0.005^∗^	0.007^∗^
Age (years)	4.6 ± 1.2	5.3 ± 1.2	4.7 ± 1.0	0.310	—	—	—
Age (months)	59.9 ± 15.3	68.9 ± 16.5	63.1 ± 13.4	0.318	—	—	—
Percentile rank	3.0 ± 2.0	0.1 ± 0.0	31.3 ± 23.6	0.000^∗^	0.000^∗^	0.000^∗^	0.000^∗^

^∗^ *p* < 0.05.

**Table 6:** Differences among subtypes based on Functional Independence Measure for Children (WeeFIM) scores.

	Subtype			*p* value	*p* value Subtype		
	I	II	III		I-II	I-III	II-III
Self-care							
Eating	5.7	5.6	6.4	0.110	—	—	—
Grooming	5.6	5.4	6.2	0.310	—	—	—
Bathing	4.2	3.7	5.5	0.030^∗^	1.000	0.074	0.113
Dressing (upper body)	5.3	4.7	6.4	0.046^∗^	1.000	0.151	0.070
Dressing (lower body)	5.7	4.9	6.5	0.035^∗^	0.775	0.177	0.046^∗^
Toileting	5.4	4.6	6.2	0.161	—	—	—

Sphincter control							
Bladder management	5.7	6.3	6.1	0.757	—	—	—
Bowel management	5.4	5.4	6.2	0.468	—	—	—
Transfers							
Chair	6.4	6.6	6.8	0.452	—	—	—
Toilet	6.1	6.0	6.7	0.213	—	—	—
Tub	5.7	5.3	6.2	0.089	—	—	—
Locomotion							
Walk	6.6	6.9	6.8	0.579	—	—	—
Stairs	6.0	5.7	6.5	0.125	—	—	—

Communication							
Comprehension	4.8	4.3	5.8	0.002^∗^	0.416	0.011^∗^	0.013^∗^
Expression	4.3	4.0	5.6	0.011^∗^	1.000	0.030^∗^	0.026^∗^
Social cognition							
Social interaction	4.0	4.0	5.1	0.058	—	—	—
Problem solving	3.3	3.6	4.5	0.078	—	—	—
Memory	4.7	4.9	5.5	0.163	—	—	—

Motor subscore	73.7	71.0	82.5	0.072	—	—	—
Cognitive subscore	21.1	20.7	26.5	0.010^∗^	1.000	0.025^∗^	0.035^∗^
Total score	94.9	91.7	109.0	0.018^∗^	1.000	0.033^∗^	0.100

^∗^ *p* < 0.05.

## Data Availability

The datasets for the current study are available from the corresponding author upon reasonable request.
